# VPA/PLGA microfibers produced by coaxial electrospinning for the treatment of central nervous system injury

**DOI:** 10.1590/1414-431X20208993

**Published:** 2020-04-09

**Authors:** K.P. Reis, L.E. Sperling, C. Teixeira, L. Sommer, M. Colombo, L.S. Koester, P. Pranke

**Affiliations:** 1 Laboratório de Hematologia e Células-tronco, Faculdade de Farmácia, Universidade Federal do Rio Grande do Sul, Porto Alegre, RS, Brasil; 2 Laboratório de Células-tronco, Instituto de Ciências da Saúde, Universidade Federal do Rio Grande do Sul, Porto Alegre, RS, Brasil; 3 Programa de Pós-Graduação em Ciências Biológicas: Fisiologia, Universidade Federal do Rio Grande do Sul, Porto Alegre, RS, Brasil; 4 Curso de Medicina, Escola da Saúde, Universidade do Vale do Rio dos Sinos, São Leopoldo, RS, Brasil; 5 Programa de Pós-Graduação em Ciências Farmacêuticas, Universidade Federal do Rio Grande do Sul, Porto Alegre, RS, Brasil; 6 Instituto de Pesquisa com Células-tronco, Porto Alegre, RS, Brasil

**Keywords:** Coaxial electrospinning, VPA, Spinal cord injury

## Abstract

The central nervous system shows limited regenerative capacity after injury. Spinal cord injury (SCI) is a devastating traumatic injury resulting in loss of sensory, motor, and autonomic function distal from the level of injury. An appropriate combination of biomaterials and bioactive substances is currently thought to be a promising approach to treat this condition. Systemic administration of valproic acid (VPA) has been previously shown to promote functional recovery in animal models of SCI. In this study, VPA was encapsulated in poly(lactic-co-glycolic acid) (PLGA) microfibers by the coaxial electrospinning technique. Fibers showed continuous and cylindrical morphology, randomly oriented fibers, and compatible morphological and mechanical characteristics for application in SCI. Drug-release analysis indicated a rapid release of VPA during the first day of the *in vitro* test. The coaxial fibers containing VPA supported adhesion, viability, and proliferation of PC12 cells. In addition, the VPA/PLGA microfibers induced the reduction of PC12 cell viability, as has already been described in the literature. The biomaterials were implanted in rats after SCI. The groups that received the implants did not show increased functional recovery or tissue regeneration compared to the control. These results indicated the cytocompatibility of the VPA/PLGA core-shell microfibers and that it may be a promising approach to treat SCI when combined with other strategies.

## Introduction

Electrospun nanofibers are regarded as a very promising extracellular matrix‐mimicking system and an effective delivery system of biomolecules, which can provide physical support for cellular growth to modulate tissue regeneration (1,2).

Spinal cord injury (SCI) is a major cause of paralysis. This lesion damages axonal pathways, interrupting synaptic transmission between the brain and spinal cord and subsequently altering motor, sensory, and autonomic functions below the level of injury (3). The complex pathophysiology of SCI may explain the current lack of an effective therapeutic approach for the regeneration of damaged neuronal cells and the recovery of motor function (4). There is no effective clinical treatment to date for this condition and current treatment focuses on stabilization and prevention of further damage. For this reason, many studies propose the use of biomaterials to repair the broken neuronal circuitry of the injured spinal cord. Implantable biomaterials can be mainly used to regenerate a damaged area of the spinal cord, bridge the formed gap, and act as support for axonal re-growth (5).

Previous studies have demonstrated that systemic administration of valproic acid (VPA) improved locomotor function after SCI (6–8). In addition, VPA exerts an anti-inflammatory effect (9), reduces cell death of motor neurons (10) and cellular apoptosis (11), attenuates demyelination and axonal loss, preserves the oligodendrocytes and neurons (6), increases neurite outgrowth (12), reduces the cystic cavity (8), and increases expression of neuronal progenitor cells in the spinal cord (13).

The intraperitoneal injection of VPA has some disadvantages. The injection method involves repeated punctures, in general twice a day for seven days (6,7,11), which can result in pain and infections (14). Therefore, biomaterial-based drug delivery systems such as microfibers present an additional platform to locally deliver VPA and therefore promote spinal cord tissue repair.

Electrospinning is currently one of the simplest methods to produce micro/nanofiber scaffolds. Coaxial electrospinning is a modification of this classical procedure, which promotes production of fibers with a core-shell structure and highly varied compositions (15). It is possible to encapsulate a number of agents such as cells, growth factors, small molecules, and nanoparticles into the fibers (16). Electrospun fibers have been used extensively as potential scaffolds in SCI tissue engineering (14,17). A wide range of natural and synthetic polymers can be electrospun. Poly(lactic-co-glycolic acid) (PLGA) has been used in many tissue engineering applications due to its biodegradability and biocompatibility (16).

To our knowledge, this is the first study to demonstrate the potential of encapsulating VPA in electrospun microfibers and its application in SCI repair.

## Material and Methods

### Preparation of microfiber scaffolds

The scaffolds were produced by the coaxial electrospinning technique. The shell solution consisted of 18% PLGA (Mw ≅50–75 kg/mol; 75:25 lactide/glicolide; PURAC Biochem BV, The Netherlands) in 1,1,1,3,3,3-hexafluoro-2-propanol (Sigma-Aldrich, USA) and chloroform (3:1) (Dinâmica, Brazil). The core of the fibers contained 25 μg/mL VPA sodium salt (VPA, Santa Cruz Biotechnology, USA), 10% polyethylene glycol (Mw≅ 20,000; Sigma) for increasing the viscosity, and 2% bovine serum albumin (BSA; Sigma) for increasing the stability of the VPA diluted in water. The prepared solutions were then delivered to the outer and inner coaxial needle at 2.0 and 0.2 mL/h feeding ratios, respectively, with a programmable syringe pump. The applied voltage was in the range of 16–25 kV and the distance between the needle and the collector plate was 15 cm (18). The fibers were collected on an aluminum collecting plate during a 30 min period. The coaxial electrospinning procedure was performed at 22°C with 45% controlled air humidity within the electrospinning apparatus (IME Technologies, The Netherlands). The control core-shell PLGA fibers were produced by the same procedure cited above, but without adding VPA to the core solution.

### Scaffold characterization

The scaffolds were characterized for their morphology, hydrophilicity, and mechanical properties. The average diameter of the fibers was determined using the software ImageJ 1.383 (NIH, USA) by measuring 30 fibers from each of the images obtained by scanning electron microscopy (SEM) (n=30).

#### Morphological analysis

The morphology of the electrospun scaffolds was analyzed by SEM (JSM 6060, USA). The collected fibers were dried overnight to evaporate the residual solvent and were then gold-coated using a sputter coater (Bal-Tec SCD 050, Leica, USA) prior to observation by a SEM operating at an accelerating voltage of 10 kV. The fiber diameter was evaluated by measuring 30 fibers in three different fields of the same sample in triplicate, resulting in 270 fibers analyzed using ImageJ software.

#### Laser scanning confocal microscopy (LSCM)

LSCM (Olympus Fluoview FV1000, USA) was used to visualize the distribution of VPA in the microfibers, and to do so, the core solution used for electrospinning was mixed with fluorescein (Sigma).

#### Static water surface contact angle

The contact angle was measured using a Drop Shape Analyzer (Krüss, Germany). A volume of approximately 5 µL of deionized water was dropped on the surface of the electrospun scaffolds and contact angle values were calculated. To prepare samples for water contact angle measurement, the microfibers were collected during a period of 10 min by the coaxial electrospinning process (n=3).

#### Mechanical properties tests

Young's modulus, maximum load (tensile stress, and maximum elongation (ultimate strain, %) were determined by dynamic mechanical analysis (DMA) in a Q800AT DMA instrument (TA Instruments, USA) equipped with a tension film clamp in the DMA controlled force mode. Scaffolds of 25×7 mm were analyzed with a ramp force of 0.5 N/min until 18 N maximum load, under 0.005 N static load at a constant temperature (37°C). The stress-strain curves were recorded and the tensile stress at maximal load was obtained from these data for each sample. The TA Universal Analysis software (TA Instruments) was used for drawing the diagrams and analyzing the results. Young's modulus of the samples was determined as the slope of the straight-line stress-strain relationship (n=3).

### *In vitro* release of VPA from VPA/PLGA microfibers

The electrospun scaffolds were placed in 7 mL of phosphate buffered saline (PBS) with 1% penicillin/streptomycin (Sigma-Aldrich). The incubation was performed at 37°C in the presence of 5% CO_2_. At appropriate intervals of 1, 6, 24 h, and 3, 5, and 10 days, 1 mL of the supernatant was removed and replenished with an identical volume of fresh buffer. The VPA concentrations were determined by high performance liquid chromatography (HPLC). The sample was filtered through a 0.45-µm membrane filter (Millipore, USA). The samples were acidified to pH 4 with hydrochloric acid (1 M). The amount of VPA released was determined using HPLC (19). The HPLC apparatus consisted of HPLC Prominence device (Japan) equipped with FCV-10 AL system controller, LC-20 AT pump system, SIL-20A automatic injector, and SPD-M20A detector. VPA was analyzed using a Kinetex^®^ 5 µm C18 100 Å, LC column of 150×4.6 mm. The mobile phase was a 55:45 (v/v) mixture of 0.05% trifluoroacetic acid (Tedia, USA) in water and acetonitrile. The injection volume was 20 µL and the HPLC system was operated at an isocratic flow of 1.0 mL/min, with detection at 210 nm. A stock solution of VPA (20 mg/mL) was prepared in methanol. The stock solution was then diluted with PBS acidified to pH 4 with hydrochloric acid (1 M) to give a series of working standard solutions for the calibration curve (10–200 µg/mL). The results are reported as means±SD (n=3).

### PC12 cell culture

Pheochromocytoma 12 (PC12) cells were cultivated in high glucose DMEM (Sigma) supplemented with 15% FBS (Gibco, USA), 5% horse serum (Laborclin, Brazil), and 1% penicillin/streptomycin (Sigma). The cells were maintained at 37°C in a humidified incubator with 5% CO_2_, and the culture medium was changed every other day. The scaffolds were cut to fit into the wells of a 24-well plate and fixed with silicon O-rings. All the samples were sterilized for 1 h under UV light before cell seeding. A total of 10,000 PC12 cells were seeded on each scaffold.

#### SEM analysis of cell growth on scaffolds

After 3 and 7 days in culture, the cell-scaffold constructs were rinsed twice with PBS, fixed with 4% paraformaldehyde (Sigma) for 20 min and dehydrated in graded series of alcohol (25, 40, 60, 75, 85, 100%) for 15 min each. After drying, the scaffolds were coated with gold (Bal-Tec SCD 050) and observed. A scanning electron microscope (Carl Zeiss EVO50, Germany) was used to observe the morphology of the cells on the microfibers from two different experiments at an accelerating voltage of 10 kV.

#### Analysis of the cell morphology by confocal microscopy

After 3 and 7 days in culture, all the scaffolds were rinsed with PBS, fixed in 4% paraformaldehyde for 20 min, and permeabilized with 0.1% Triton-X100. The cells were then stained with 20 μg/mL rhodamine-phalloidin and 0.5 μg/mL (4',6-diamidino-2-phenylindole) DAPI (Life Technologies, USA), and washed 3× with PBS. Following this, images were taken by Z-stack scanning and 3D reconstruction of an Olympus Fluoview FV1000 confocal microscope.

### VPA bioactivity

The PC12 cell lineage was used to evaluate the bioactivity of VPA. It is expected that VPA inhibits the proliferation of pheochromocytoma cells (20). For this reason, the scaffolds were cut to fit into the wells of a 24-well plate and fixed with silicon O-rings. The material was sterilized by UV light for 1 h before cell seeding. PC12 cells at 10,000 cells per well were seeded onto the scaffolds at 37°C with 5% CO_2_. The culture medium was high glucose DMEM (Sigma) supplemented with 15% FBS (Gibco), 5% horse serum (Laborclin, Brazil), 1% penicillin/streptomycin (Sigma), and 0.1% amphotericin (Sigma). The WST-8 assay was used to determine the impact of VPA on the viability cells (n=3).

After 3 and 7 days, the cells were treated with WST-8 (4-[3-(2-methoxy-4-nitrophenyl)-2-(4-nitrophenyl)-2*H*-5-tetrazolio]-1,3-benzene disulfonate sodium salt) for 2 h. This assay is based on the conversion of the tetrazolium salt WST-8 to highly water-soluble formazan by viable cells. After the incubation period, the absorbance of the culture media with WST-8 was measured at 420 nm using a plate reader. The percentage of viable cells was calculated using the optical density of the control and treated cells.

Two experimental groups were used: control PLGA scaffold, cells were cultivated on electrospun PLGA core-shell fibers without VPA, and VPA/PLGA scaffold, cells were cultivated on electrospun PLGA core-shell fibers with VPA in the core of the fibers. A control group, which consisted of cells directly cultivated on the well, was also evaluated by WST-8 assay.

### *In vivo* tests

A total of 18 male Wistar rats aged 2 months (250-300 g body weight) were obtained from the Animal House of the Instituto de Ciências Básicas da Saúde da Universidade Federal do Rio Grande do Sul. They were maintained in a temperature-controlled room (21±2°C) on a 12-h light/dark cycle, with food and water available *ad libitum*. All the procedures were in accordance with the Guide for the Care and Use of Laboratory Animals adopted by the National Institutes of Health (USA) and with the Federation of Brazilian Societies for Experimental Biology. The study was approved by the Research Ethics Committee of the University (#28079). The animals were randomly divided into three experimental groups: SCI (laminectomy followed by SCI), PLGA scaffold (SCI with implanted PLGA scaffold), and VPA/PLGA scaffold (SCI with implanted VPA/PLGA scaffold).

#### Spinal cord injury and scaffold implantation in rats

Spinal cord injury by right-side hemisection was performed, as described previously with some modifications (21). All the animals were anesthetized by an intraperitoneal (*ip*) injection of a mixture of xylazine (5-10 mg/kg) and ketamine (75-100 mg/kg). A longitudinal incision was made and a laminectomy was performed at two vertebral segments, T9-T10. The spinal cord was then hemisected at T10 on the right side by placing a 28-gauge needle dorsi-ventrally at the midline of the cord and pulling it laterally to ensure a complete hemisection. The scaffolds, with a diameter of 2 mm and a thickness of approximately 300 µm, were carefully placed into the hemisected gap immediately after the SCI. Subsequently, the fascia, musculature, and skin were sutured. Antibiotic (10 mg/kg enrofloxacin; Bayer, Brazil) was administered *ip* for 5 days after the procedure to prevent infection, and analgesic (10 mg/kg tramal; Pfizer; USA) was administered to prevent pain, followed by two drops of baby Tylenol twice a day for 5 days.

#### Locomotor activity assessment

Hind limb locomotor function was assessed with the Basso, Beatie and Bresnahan (BBB) scale. Each score represents a distinct motor functional state from 0 (complete paralysis) to 21 (normal mobility) through joint movements, stepping ability, coordination, and trunk stability. Evaluation began 2 days after injury and was repeated weekly until the sixth week after SCI and was performed in an open field by two separate observers.

#### Flow cytometry analysis

Six weeks after the implantation, the animals’ spinal cords were isolated. A 1-cm fragment was collected, including the epicenter of the lesion and equal rostral end caudal portions. The non-degraded PLGA membranes were removed and the tissue was mechanically and enzymatically dissociated with trypsin (Sigma-Aldrich). The cell suspension was fixed for 30 min with 4% paraformaldehyde and subsequently blocked for 30 min with 3% BSA in PBST. After blocking for 20 min with 3% BSA in PBS with 0.1% Triton X-100, the cells were incubated with primary antibodies, including anti-GFAP (DAKO; 14.5 μg/mL), anti-βIII tubulin (Millipore, 05559), anti-nestin (Santa Cruz, SC-33677, 1 μg/mL), and anti-CD68 (Millipore, MAB 1435). The cells were washed twice with PBS1X and incubated for 1 h with the secondary antibody Alexa-fluor 488 anti-mouse or anti-rabbit (10 μg/mL, Thermo Fisher Scientific, USA) at 37°C. Negative controls (samples incubated only with the secondary antibody) were included for setting up the machine voltages and to determine the negative population. The cells were analyzed using a FACSAria III cytometer (Becton Dickinson Biosciences, USA), equipped with a 488 nm argon laser and the FACSDiva 6.0 software. An average of 5×10^4^ events was analyzed.

### Statistical analysis

The experiments were done in triplicate unless otherwise stated and all the data are reported as means±SD. Statistical analysis was performed using *t*-test and one-way ANOVA, followed by the Bonferroni *post-hoc* test. A P value of less than 0.05 was considered statistically significant. Statistical analysis was performed using GraphPad Prism 5 for Windows (USA).

## Results

### Characterization of the electrospun scaffolds

The fiber morphology, as seen by SEM, is shown in Figure 1. Both groups of electrospun microfibers showed a smooth and bead-free surface with uniform diameters (Figure 1A and C). It can be concluded that VPA was incorporated into the electrospun PLGA microfibers without modifying the fiber shape. Image analysis showed that the average fiber diameters for PLGA and VPA/PLGA were 2.18±0.74 μm and 2.00±0.61 μm, respectively, with no significant difference between the two groups.

**Figure 1:** Scanning electron microscopy images showing the morphology of the microfibers. **A**, Poly(lactic-co-glycolic acid) (PLGA) coaxial electrospun fibers with an average diameter of 2.18±0.74 μm and (**C**) valproic acid (VPA)/PLGA coaxial microfibers with an average diameter of 2.0±0.61 μm. **B** and **D** show the corresponding histograms of the fiber diameter distribution. Scale bars: 10 µm.

To provide evidence of the successful incorporation of VPA into fibers, fluorescein was loaded as the core solution and then its distribution inside the nanofiber was observed by confocal microscopy. Figure 2A shows the presence of green fluorescence in the fibers and the uniform distribution, suggesting the incorporation of the substance in the core.

**Figure 2:** **A**, Confocal fluorescence microscopy image of the core-shell electrospun microfibers using fluorescein in the core (scale bar: 5 μm). **B** and **C,** images from contact angle measurement of PLGA (129.7±0.01°) and VPA/PLGA 127.0±1.80° scaffolds, respectively (n=3).

Hydrophilicity of the electrospun microfiber scaffolds was measured by water contact angle. For the PLGA microfibers, the contact angle was 129.7°±0.01, which was similar to that of 127.0°±1.80 obtained from the VPA/PLGA core-shell microfibers (Figure 2B and C). The addition of VPA did not modify the water contact angle of the scaffolds.

### Mechanical properties

The mechanical properties of the coaxial microfibers were evaluated according to the following categories: Young's modulus (MPa), tensile stress at yield (MPa), and tensile strain at maximum (%). Table 1 shows the results obtained from the respective measurements. The spinal cord presents specific viscoelastic characteristics with specific mechanical properties and therefore the mechanical properties of the microfibers should be similar to the neural tissue. The scaffolds should provide sufficient mechanical support for neural regeneration.

**Table 1:** Young's Modulus (MPa), maximal elongation (%) under the applied force, and the maximal load (MPa).

Sample	Young's modulus (MPa)	Maximal elongation (%)	Maximal load (MPa)
PLGA	1.437±1.11	177.83±13.97	0.538±0.06
VPA/PLGA	1.758±0.94	204.03±8.15	0.693±0.12

Data are reported as means±SD (n=3). PLGA: poly(lactic-co-glycolic acid); VPA: valproic acid.

### *In vitro* release of VPA and bioactivity

The VPA cumulative release from the scaffolds incubated in PBS, pH 7.4 at 37°C was analyzed by HPLC, as shown in Figure 3. The release profile showed an initial burst release during the first day, followed by a gradual sustained release.

**Figure 3:** Cumulative release profile of valproic acid (VPA) from core-shell fibers determined by high performance liquid chromatography. Data are reported as means and SD. The experiments were performed in triplicate.

### Cytocompatibility of VPA-PLGA core-shell fibers

The cell morphology, spreading, and viability of rat PC12 cells on the microfibers were analyzed. The PC12 cells were used because of their ectodermal origin. As shown in Figure 4, the scaffolds had good biocompatibility and favored PC12 cell attachment, spreading, and proliferation, 3 and 7 days after seeding. PC12 adhered well to the surface of the scaffolds and showed good integration with the fibers (Figure 4 A and B). No morphological differences were observed between the cells cultivated on the PLGA fibers and VPA/PLGA fibers (see Figure 4). The Wst-8 assay showed that cell proliferation on all the scaffolds increased with culture time (Figure 5). When compared to the control cells cultivated directly on the culture plate, a reduction in cell viability was observed in the cells cultivated on the PLGA and PLGA/VPA scaffolds. Moreover, after 7 days in culture, the VPA/PLGA significantly inhibited the growth of the PC12 cells (Figure 5).

**Figure 4:** Scanning electron microscopy and fluorescence microscopy images of PC12 cells cultivated on the poly(lactic-co-glycolic acid) (PLGA) scaffold (**A** to **D**) and valproic acid (VPA)/PLGA scaffold (**E** to **H**) after 3 and 7 days in culture (n=2). In red are the actin filaments stained by rhodamine phalloidin; in blue, cell nuclei stained by DAPI. The cells attached and spread on the biomaterials. Scale bars: 10 µm.

**Figure 5:** Analysis of cell viability on the poly(lactic-co-glycolic acid) (PLGA) and valproic acid (VPA)/PLGA scaffolds by WST-8 assay. The absorbance value (405 nm) was measured at 3 and 7 days in culture. Data are reported as means±SD (n=3). *P<0.05, one-way ANOVA.

### *In vivo* results

#### Analysis of locomotor recovery after SCI using the BBB scale

Adult rats were submitted to a hemisection lesion of spinal cord, which led to the paralysis of the ipsilateral member. BBB scoring is a common method to assess locomotor function of rats after SCI. Two trained investigators who were blind to the experimental conditions scored the locomotion recovery in an open field according to the BBB scale. The BBB scores, which are shown in Figure 6, demonstrated that there was no significant difference at any of the weekly time points between the control and scaffold groups.

**Figure 6:** Basso, Beatie and Bresnahan (BBB) open-field walking scores for the spinal cord injury (SCI, control), poly(lactic-co-glycolic acid) (PLGA), and valproic acid (VPA)/PLGA groups on the ipsilateral, lesioned side (n=6 animals/group). Data are reported as means±SD.

#### Analysis of cellular markers by flow cytometry

After the injury, the cell suspensions obtained from 1-cm long spinal cord tissue containing the epicenter of the lesion were immunostained with antibodies specific to neurons (TUJ), astrocytes (GFAP), and macrophages (CD68). Figure 7 shows the percentage of cells positive for βIII-tubulin, nestin, GFAP, and CD68 expression. No significant difference in the number of the expressing cells between the groups was observed.

## Discussion

SCI can cause clinically irreversible disability and result in a high level of comorbidity. In adult mammals, the central nervous system exhibits insufficient regeneration capacity; therefore, various therapeutic strategies have been applied to improve the regeneration of injured spinal cord. Biomaterial-based scaffolds have been designed to provide mechanical support and deliver biochemical signals to modulate specific cellular responses (16). Thus, in the present study, core-shell microfibers of PLGA encapsulating VPA were produced. The scaffold of randomized coaxial fibers was implanted at the site of the hemisected spinal cord to create a bridge that could span over the spinal cord injury site as well as provide neuroprotection through the local release of VPA. The SCI animals that received the scaffold implant displayed modest gains in functional recovery. This is the first study to demonstrate the potential of encapsulating VPA in electrospun microfibers and its application in SCI repair.

Coaxial electrospinning resulted in samples with continuous and smooth cylindrical morphology, randomly oriented fibers with fairly uniform diameter and without any beads (Figure 1), which indicated the stability of the electrospinning process (22). Analysis of the contact angle showed that there was no significant difference in the values of the coaxial microfibers compared with the uniaxial PLGA fibers. Moreover, the contact angle value was similar to that reported by previous studies (23). This result indicated that there was no extravasation of the core content of the fibers (24). Bilston and Thibault (25) reported that the average Young's modulus (MPa) of spinal cord tissue was 1.37±0.39 MPa. Comparing the value of the tissue with the value obtained for the VPA/PLGA fibrous scaffold, it can be concluded that the produced microfibers had sufficient tensile stress to be utilized as a biomaterial for the treatment of SCI.

VPA was incorporated into the PLGA microfibers without modifying the morphology and fiber shape (Figure 1). A burst release of the VPA in the first 6 h was observed, which comprised around 80% of the encapsulated substance (Figure 3). The burst effect is functional for the treatment of primary SCI, contributing to the reduction of the cascade of secondary events and attenuation of a specific cellular response (4). Moreover, the core-shell fibers present a thinner sheath layer and the porous structure of the fiber surface may allow for higher water adsorption and for more drug molecules to diffuse out of the core into the surrounding media (24).

In order to test the biocompatibility of the PLGA and VPA/PLGA core-shell fibers, the PC12 cell line was used and their proliferation and adhesion onto the scaffold was analyzed. PC12 cells are derived from a tumor (pheochromocytoma) of the rat adrenal medulla. Given the neural origin of the adrenal medulla, these cells are widely used as a model in neurophysiological and neuropharmacological studies (26). All the experimental groups were able to support cell attachment and growth (Figure 4). The control group presented greater absorbance compared with the other groups, representing a larger number of cells in the wells of the plastic plates (cell culture control). Such a result was expected because cultivating cells in plastic wells is the conventional procedure, and a high viability on plastic has already been observed in previous studies (27,28). The cells also presented similar viability at day 3, indicating that there were no differences in the cell ability in terms of the cells attaching to the biomaterials. However, on day 7, PC12 cell viability on the VPA/PLGA microfibers group was significantly lower than that of the PLGA group. Adler and collaborators (20), who studied the effect of VPA on the growth of PC12 cells, demonstrated that the treatment of PC12 cells with VPA inhibited the growth of this cell type by activation of cellular apoptosis, thereby making VPA a drug candidate for the treatment of pheochromocytomas. The present results are therefore indicative of the maintenance of VPA bioactivity after its encapsulation in microfibers.

In order to test the effect of VPA/PLGA core-shell fibers on neural regeneration, a lateral hemisection SCI rat model was used. After lesioning, the motor behavior of the animals was analyzed by open field BBB scoring. According to BBB analyses, the function of hind limb ipsilateral to the injury was severely impaired after the operation; meanwhile the contra-lateral hind limb was inevitably affected. There was no significant difference in functional recovery between the experimental scaffolds and control groups (Figure 6). Previous study showed that systemic administration of VPA by injecting an initial bolus of VPA immediately after injury and maintaining an injection frequency for a certain period increased motor recovery after SCI (7). This showed that the therapeutic effect of VPA varied with the model used and gravity of SCI. Further studies should increase the amount of encapsulated VPA, since no obvious motor recovery was observed in this experiment. The use of other biodegradable polymers as a shell could represent another possibility. Polycaprolactone, for example, has a slower degradation rate, which would lead to a longer and more sustained release of VPA. It is also possible that the number of animals used in each group (n=6) was insufficient to demonstrate statistical significance.

Flow cytometry analyses revealed that βIII-tubulin expression was not altered by the presence of the VPA/PLGA scaffold. The scaffold therefore had no adverse effect on the neural cell populations in the injured spinal cord, indicating that it is safe for use in the treatment of SCI. Although VPA was shown to improve neuroprotection and neurogenesis (13), no significant increase in neural or neuroprogenitor cells was detected by flow cytometry.

Furthermore, there was no difference between the groups for CD68 expression. This is indicative that the scaffolds did not induce inflammatory responses at the lesion site. The expression of the astrocyte specific marker GFAP was reduced in the PLGA and VPA/PLGA scaffolds compared with the control lesion group at 6 weeks after lesion (Figure 7). This result indicated a reduction in glial scaring at the lesion site in these indicated groups, which is in accordance with the study of Darvish and collaborators, which demonstrated that treatment with VPA reduces GFAP expression in SCI rats (8).

**Figure 7:** Analysis of expression of βIII-tubulin, Nestin, GFAP, and CD68 by flow cytometry for the control, poly(lactic-co-glycolic acid) (PLGA), and valproic acid (VPA)/PLGA groups. Results are reported as percentage of positive cells (n=4/group). Data are reported as means±SD.

In this study, core-shell microfiber scaffolds with encapsulated VPA were successfully produced by coaxial electrospinning. The scaffolds showed good biocompatibility, as seen by the *in vitro* tests. PC12 cells were able to attach and proliferate onto the scaffolds. In addition, when the scaffolds were implanted into the hemisected spinal cord of rats they did not demonstrate negative effects on the neural cell populations and did not cause inflammatory responses at the lesion site. This study could also be considered a basis for further development of VPA/PLGA scaffolds as a suitable substrate to be combined with other strategies.
